# Impact of Health-Promoting Lifestyle Education Intervention on Health-Promoting Behaviors and Health Status of Postmenopausal Women: A Quasi-Experimental Study from Sri Lanka

**DOI:** 10.1155/2019/4060426

**Published:** 2019-12-16

**Authors:** Nirmala Rathnayake, Gayani Alwis, Janaka Lenora, Sarath Lekamwasam

**Affiliations:** ^1^Department of Nursing, Faculty of Allied Health Sciences, Matara, University of Ruhuna, Sri Lanka; ^2^Department of Anatomy, Faculty of Medicine, University of Ruhuna, Matara, Sri Lanka; ^3^Department of Physiology, Faculty of Medicine, University of Ruhuna, Matara, Sri Lanka; ^4^Population Health Research Centre, Department of Medicine, Faculty of Medicine, University of Ruhuna, Matara, Sri Lanka

## Abstract

Health promotion through lifestyle education is an important measure to enhance health status of postmenopausal women (PMW). This study evaluated the effectiveness of health-promoting lifestyle education intervention (HPLEI) on adhering to health-promoting behaviors (HPB) and enhancing the health status in a group of Sri Lankan PMW. A quasi-experimental study was conducted with randomly selected, sociodemographic status matched, 72 PMW from two geographically separated areas in Galle District, Sri Lanka, allocated as experimental (*n* = 37, 54.6 ± 4.5 years) and control (*n* = 35, 56.5 ± 3.4 years) groups. Education intervention focused on postmenopausal health management including lifestyle modifications was performed only for the experimental group during 8 weeks, and a health education package was provided. The control group was not given any planned education programme. Both groups were followed up for a 6-month period. HPB and menopausal symptoms severity were evaluated by validated Health Promoting Lifestyle Profile-II and Menopause Rating Scale, respectively. Anthropometric adiposity indices (AAIs) including weight, body mass index (BMI), waist (WC) and hip (HC) circumferences, and waist to hip ratio (WHR); cardiovascular disease risk indicators (CVDRI) including systolic blood pressure (SBP), diastolic blood pressure (DBP), fasting blood sugar (FBS), total cholesterol and triglycerides, muscle strength; hand grip strength (HGS) and physical performance (PP); gait speed (GS) were measured. All parameters were evaluated before the intervention (baseline) and after follow-up of 6 months. All evaluated parameters were not different between experimental and control groups (*p* > 0.05) at the baseline. In the follow-up evaluation, HPB (*p* < 0.001), menopausal symptom scores (*p* < 0.001), AAI (*p* < 0.001), CVDRI (SBP, DBP, and FBS) (*p* < 0.05) and HGS and GS (*p* < 0.001) were significantly improved in the experimental group but not in the control group. Health education intervention focused on health-promoting lifestyle modifications is effective in improving the adherence to HPB and enhances the health status in PMW. This provides positive impact in lifestyle medicine.

## 1. Background

Health promotion is “the fundamental strategy in health care that implies changes in behavior and the adoption of patterns that promote good health in order to improve the quality of life (QOL) of the people.” [1] The main goal of health promotion is achieving healthy lifestyle behaviors [2] known as “health-promoting behaviors” (HPB). HPB are important for the empowerment of individuals for achieving optimum health and preventing diseases [3–5].

Menopause is a significant landmark in the reproductive life of women, and hormonal changes at menopause create a multitude of structural and functional changes in postmenopausal women (PMW). These include menopausal symptoms [6], changes in anthropometric adiposity indices (AAI) [7], cardiovascular disease risk indicators (CVDRI) [8], muscle strength, and physical performance (PP) [9]. These changes have the potential to progress to debilitating chronic diseases and functional disabilities [10–14] in later life.

Unhealthy lifestyles such as lack of physical activities, improper dietary practices, and poor stress relief aggravate the consequences of hormonal changes in PMW leading to impaired QOL [10, 14]. Therefore, educating PMW on suitable lifestyle modifications is a need in this period of life [15]. Regular training or education programs on healthy lifestyle are vital to promote health in general and QOL [16, 17]. Positive lifestyle changes such as physical activity and dietary modifications have clear benefits on many aspects of life in PMW, including physical and emotional changes, sleep, and cardiovascular health [18].

Health education improves health literacy and develops life skills. In educating PMW, it is important to identify methods which are effective, practical, and affordable. Furthermore, they should be able to accommodate such education programmes in their daily routine work. Despite the clear benefits which education programmes have shown in previous studies, there is a paucity of studies conducted in Sri Lanka on this vital area. The average age of a Sri Lankan women attaining menopause is between 49 and 51 years. Considering the female life expectancy of 78 years, a woman has to spend approximately three decades in her life in the postmenopausal period. Therefore, overall health and well-being of PMW have become a major global public health concern and need strict attention with proper guidance to enhance the health status. Hence, this intervention study was designed to evaluate the effectiveness of a health-promoting lifestyle education intervention (HPLEI) on adhering to HPB and enhancing health status in a group of PMW in Sri Lanka.

## 2. Materials and Methods

### 2.1. Study Design, Participants, and Setting

This quasi-experimental study was designed, as a part of a main study “Effects of menopause on bodily structure, functions and physical health,” conducted at the Faculty of Medicine, University of Ruhuna, Sri Lanka. Among the 18 public health midwifery (PHM) division (the smallest primary health care unit of the country) of Bope-Poddala medical officer of health (MOH) area, Galle, 5 PHM divisions were selected randomly for the main study with 166 PMW. Of the 5 PHM divisions, 2 divisions were selected randomly for the “experimental group” and another 2 geographically separated PHM divisions were selected randomly for the “control group” to minimize the contamination. One PHM division was excluded from this intervention. The two groups were matched for age, age at menopause, time since menopause, and sociodemographic status.

Sample size for the HPLEI was decided by comparing the QOL before and after an education intervention among PMW in Iran [19], using the formula *N* = (*Z*_*α*/2_+*Z*_*β*_)^2^ ∗ (*σ*1^2^ + *σ*2^2^)/(*μ*1 – *μ*2)^2^. After adding 10% for dropouts, the minimum required sample size was 42 PMW in each group. Based on the inclusion and exclusion criteria, 42 women were allocated to the experimental group and 38 women were allocated to the control group.

Postmenopausal status was considered on self-stated menstrual history based on the classification of Stages of Reproductive Aging Workshop (STRAW) [20] which is the cessation of menstruation within the previous 12 months after last menstruation. Women on hormone replacement therapy (HRT) or with noncommunicable diseases (NCDs), disorders related to musculoskeletal and nervous system, and gait or balance problems were excluded. Also women aged 60 years or more or premature menopause (menopausal age <40 years) and menopause secondary to surgery or drug therapy were excluded from the basic screening study.

Consenting women educated at least up to grade 5, time since menopause ≥2 to ≤7 years, and physically and mentally healthy were included in the current study.

During the study, in the experimental group, two women died and three women were unable to participate continuously. Three women from the control group left the study due to changing residences. Finally, 37 women from the experimental group and 35 women from the control group completed the study (*n* = 72).

### 2.2. Health-Promoting Lifestyle Education Intervention

HPLEI was carried out for 8 weeks (June to July 2017), and printed health education package including lifestyle modifications was provided at the end for the experimental group. Structure of sessions, objectives, content, and teaching materials were designed by the research team with contributions from a panel including a gynecologist, physician, nutritionist, and sports physician. Teaching materials were prepared to suit the subjects without technical terms and inclusion of visual images. Timing of sessions was decided with the mutual agreement between participants and the principal investigator, and they were contacted a day prior to the scheduled session. All the sessions were conducted as a group activity led by the principal investigator, and each group comprised a maximum of 10 women. Printed materials detailing the session objectives and activities planned were provided to subjects before sessions. Duration of sessions was 1 hour: 40 minutes for educating and 20 minutes for summarizing and feedback.

HPLEI comprised menopausal symptom management, healthy diet, healthy physical exercises, and spiritual support, individualized to suit them. Available remedies for troublesome menopausal symptoms were informed. Dietary advices were individualized based on BMI and activity pattern. Daily caloric requirement was arranged as BMI <18.5 kg/m^2^: 35 kcal/kg/day; 18.5 BMI 23.9 kg/m^2^: 25–30 kcal/kg/day; and BMI >24 kg/m^2^: 20–25 kcal/kg/day [21]. Further adjustment in diet was done according to the current physical activity level. Proportion of energy was carbohydrate 55–65%; fat 20–30%; and protein 10–15%. The energy distribution of meals was breakfast 20%; lunch 40%; dinner 20%; and snacks 20%. Physical exercises were of three types: continuous walking (30 min × 5 days per week), strength training exercise for limbs (8–10 times × 3 times per day × 3 days per week), and balance training exercise (8–10 times × 3 times per day × 3 days per week). Apart from dietary advices and physical activities, they were asked to engage in relaxation exercises such as meditation for 10 minutes daily, reading books, listening to music, and engaging in religious activities.

The control group was not exposed to any planned education programme and continued as normal, however maintained the contacts with them regularly. Both groups were followed up strictly for 6-month period (August 2017–January 2018) after finishing the education sessions. All the steps of the study are shown in the flow diagram (Figure 1).

### 2.3. Evaluations of HPB and Menopausal Symptom Severities

Health Promoting Lifestyle Profile-II (HLPL-II) and Menopause Rating Scale (MRS) were used to evaluate the HPB and menopausal symptom severities, before the intervention, immediately after the intervention, and after 6 months of follow-up in women in both the groups.

HPLP-II [22] contains 52 items under six subscales (health responsibility, physical activity, nutrition, spiritual growth, interpersonal relations, and stress management) to measure the frequency of HPB. MRS assesses 11 menopausal symptoms and their severity categorized into three independent subscales (somato-vegetative symptoms, psychological symptoms and urogenital symptoms) [23]. Both HPLP-II [24] and MRS [25] have been validated locally.

### 2.4. Evaluation of AAI, CVDRI, Muscle Strength, and PP

AAI, CVDRI, muscle strength, and PP were evaluated before the intervention and 6 months after the follow-up.

AAI measured were body weight (kg), body mass index (BMI, kg/m^2^), waist (WC) and hip (HC) circumferences (cm), and waist to hip ratio (WHR). Body weight was measured to the nearest 0.1 kg while wearing light clothes, and standing height was measured without footwear and recorded to the nearest 0.1 cm with a calibrated stadiometer (NAGATA, Tainan, Taiwan). WC and HC were measured using a plastic nonstretchable tape to the nearest 0.1 cm. All the measurements were obtained adhering to standard protocols [26] by a single investigator.

CVDRI measured were systolic blood pressure (SBP), diastolic blood pressure (DBP), fasting blood sugar (FBS), and lipids: total cholesterol and triglycerides. Biochemical analyses were performed using Mindray (BA–88A) semi auto chemistry analyzer (China) with the expert technical assistance under standard laboratory conditions.

Muscle strength was measured as the hand grip strength (HGS, kg) of the dominant hand using Lafayette hand held dynamometer (Lafayette Instrument Co. Ltd, Sagamore Parkway North, USA) [27]. PP was measured as gait speed (GS, m/s), the time taken to walk the central 4 meters of an 8-meter course at usual self-selected pace. The initial and final 2 meters were excluded from the calculation to eliminate the effects of acceleration and deceleration. Both HGS and GS tests were done twice, and the average of two measurements was used for the analyses [27].

### 2.5. Statistical Analyses

For the final analysis, only 72 women were included (experimental group = 37 and control group = 35). Descriptive data are presented as means, standard deviations (SD) and for continuous data and categorical variable as frequencies and percentages (%). The data gathered in all questionnaires were analyzed with the standard guidelines provided by the respective authors and publishers [22, 23].

The differences of age and sociodemographic characteristics, AAI, CVDRI, muscle strength, and PP between experimental and control groups were compared using independent sample *t*-test and chi-square test of independence. The differences of HPB and menopausal symptoms scores within experimental and control groups in three consecutive evaluations were analyzed by the repeated measures ANOVA test with Bonferroni correction to eliminate the effect of time factor. The differences of AAI, CVDRI, muscle strength, and PP within experimental and control groups in two evaluations were analyzed by the paired sample *t*-test. Furthermore, the difference between the variables obtained at the end of 6 months of follow-up was further evaluated with one-way analysis of covariance (ANCOVA) while eliminating the effect of basic characteristics such as age and baseline values of each variable.

Statistical analyses were performed with SPSS 20.0 version, and *p* value < 0.05 was considered as statistically significant.

## 3. Results

### 3.1. Basic Characteristics of Participated Women

Basic characteristics of experimental and control groups are shown in Table 1. Age, age at menopause, time since menopause, and sociodemographic characteristics were not different between experimental and control groups (all *p* > 0.05).

There was no significant difference of HPB scores, menopausal symptom scores, AAI, CVDRI, HGS, and GS between experimental and control groups (*p* > 0.05) at the baseline (*p* values are not shown).

### 3.2. Changes of HPB, Menopausal Symptoms, and Measured Variables of Experimental and Control Groups in Three Stages of Evaluation

HPB: all the subscales scores of HPB were higher at the end of intervention when compared with baseline values (*p* < 0.001) in the experimental group. In the control group, physical activity (*p* < 0.001) and stress management scores (*p*=0.01) showed an increase while health responsibility (*p* < 0.001) and spiritual growth (*p*=0.01) showed a decrease. Nutrition and interpersonal relations remained unchanged (*p* < 0.05) (Table 2).

Menopausal symptoms: in the experimental group, all the menopausal symptom scores showed a reduction at the end of intervention (*p* < 0.001). In the control group, however, these symptom scores increased with time (*p* < 0.001) (Table 2).

AAI: all the measured AAIs showed a reduction (*p* < 0.05) in the experimental group, whereas in the control group, they were increased (*p* < 0.05) at the end of intervention (Table 3).

CVDRI: in the experimental group, SBP, DBP, and FBS showed a significant reduction at the end (*p* < 0.05). Lipids, total cholesterol and triglycerides, were also reduced; however, there was no significant difference between the two evaluations (*p* > 0.05). In the control group, SBP and DBP increased significantly at the end (*p* < 0.05). Furthermore, nonsignificant increments of FBS and total cholesterol (*p* > 0.05) and reduced triglycerides (*p*=0.06) were observed in the same evaluation (Table 3).

HGS and GS: HGS and GS improved (*p* < 0.001) at the end of intervention in the experimental group. However, in the control group, HGS did not change with time (*p*=0.52) and GS deteriorated (*p* < 0.001) (Table 3).

Between-group comparison at the end of 6 months of follow-up showed an improvement of all subscales of HPB (*p* < 0.001), all menopausal symptom subscales (*p* < 0.001) (Table 2), all AAI (*p* < 0.01), CVDRI, DBP (*p* < 0.04), FBS (*p* < 0.001), and HGS and GS (*p* < 0.01) (Table 3) in the experimental group compared to the control group during intervention.

The results did not materially change even after controlling the effect of age and baseline characteristics with the one-way ANCOVA (Tables 2 and 3).

## 4. Discussion

The current study revealed that HPLEI helped the PMW to establish good living habits, relieve from troublesome menopausal symptoms, and enhance significant improvements in AAI, CVDRI, muscle strength, and PP that will enhance the general health and QOL.

Our observations are consistent with many studies which reported the effectiveness of health education interventions focused on health-promoting lifestyle modifications. The findings of education interventions based on lifestyle modifications were effective in improving menopausal symptoms, and HPB [28–31] of PMW is consistent with that of the current study. A Chinese study also showed that a 12-week intervention helped the PMW to change HPB positively [32]. Positive effects of healthy lifestyle interventions leading to a reduction in menopausal symptoms have been observed in the experimental group of PMW in many studies [31–34]. After attending a series of health-related presentations, weight reduction [34–36] in PMW in the experimental group has been observed. Significant improvements in CVDRI such as total cholesterol, triglycerides, and FBS have been observed in PMW in few studies [35, 36]. Several studies have also shown that muscle strength and PP can be improved through lifestyle changes [37–40] in elderly women.

Positive impact of education interventions that focused on the lifestyle management in improving different aspects of health status of PMW seen consistently emphasizes the benefits of such intervention regardless of study population, duration, and intensity of the programme. Furthermore, we chose a six-month follow-up period that is reasonably a longer duration of follow-up compared to other studies [31–33], and continuous evaluation and monitoring of study participants were also helpful for observed positive outcomes.

We also observed that some HPB such as physical activity and stress management have increased in the control group too. This would be due to the fact that they may have gained knowledge from outer sources such as relatives, friends, media, and personal experience, since we could not control external stimuli, even though we did not provide any planned education to the control group.

Overall, we observed the prominent positive changes in adhering HPB and improvement of menopausal symptoms and structural changes such as AAI. However, the positive changes of HGS, GS, and CVDRI that are functional changes were not as prominent as structural changes. It is suggested that positive lifestyle changes would cause structural changes early; however, to achieve lasting functional changes, more time would be required. Furthermore, evaluation of HPB and menopausal symptoms through a self-administered questionnaire would provide exaggerated positive results; therefore, approaches such as qualitative interviews would be more beneficial in such evaluations.

Even though the literature consists of plenty of studies focused on improvement of HPB and menopausal symptoms following lifestyle education intervention, there is a paucity of literature on evaluation of AAI, CVDRI, muscle strength, and PP. Therefore, the current study would add valuable information to both local and global communities on enhancing the health status of PMW through lifestyle education and strengthen the literature related to the area of study.

The complications of menopause can be reduced if women are health literate, have necessary skills, and know how to use them effectively. This study provides a positive and effective strategy to treat and rehabilitate PMW, which is a nonhormonal, noninvasive, and low-cost management option. This would be an option for women who suffer from different problematic conditions especially for those who could not or are unwilling to use drug therapy. Therefore, healthcare professionals can educate PMW on the varying options and resources regarding menopause and well-being for behavioral changes for controlling physical and psychological problems. This programme may also offer implications for designing and implementing large-scale interventions in future in different communities in order to ensure its usefulness. Assessing the long-term effects of this intervention and health outcomes that appear in future are also recommended.

The present study is a brief education programme with a small sample size, and self-reporting of HPB and menopausal symptoms could be considered as several limitations. Despite these limitations, there are several strengths of this study. We used almost matched samples for the comparison, minimized the contacts between the two groups, used a well-designed education programme, and followed them up for comparatively lengthy periods enhancing the quality of our study. Furthermore, we were unable to find studies of similar nature done in Sri Lanka where our study will provide a platform for future research in this increasingly important area of health care.

## 5. Conclusions

The HPLEI designed for PMW was effective in improving adherence to the HPB and enhancing different aspects of health status including relieving menopausal symptoms, reducing adiposity, and improving cardiovascular functions and physical functions. This HPLEI provides positive impact of lifestyle medicine. Hence, it is recommended as a healthcare intervention in postmenopausal health management.

## Figures and Tables

**Figure 1:** Flow diagram of the health promoting lifestyle education intervention.

**Table 1:** Sociodemographic characteristics of the study participants in experimental and control groups (*n* = 72).

Characteristics	Subcategory	Experimental group (*n* = 37), mean (SD) or frequency (%)	Control group (*n* = 35), mean (SD) or frequency (%)	*p* value
Age (years)		54.6 (4.5)	56.5 (3.4)	0.06^*∗*^

Age at menopause (years)		47.9 (4.2)	49.0 (4.0)	0.24^*∗*^

Time since menopause (years)		4.6 (2.1)	5.2 (2.0)	0.30*∗*

Employment status	Employed	9 (24.3)	7 (20.0)	0.77^*∗∗*^
	Unemployed	28 (75.7)	28 (80.0)	

Civil status	Married	30 (81.1)	28 (80.0)	0.90*∗∗*
	Single or widowed or divorced	7 (18.9)	7 (20.0)	

Living companion	With husband and children	24 (64.9)	21 (60.0)	0.20^*∗∗*^
	With husband or children	9 (24.3)	5 (14.3)	
	Alone or living with others	4 (10.8)	9 (25.7)	

Education status	Primary education	5 (13.5)	10 (28.6)	0.20^*∗∗*^
	Secondary education	18 (48.6)	15 (42.9)	
	Upper secondary or tertiary education	14 (37.8)	10 (28.6)	

Monthly income	Below 20000 LKR	25 (67.6)	27 (51.9)	0.36^*∗∗*^
	Above 20000 LKR	12 (32.4)	8 (22.9)	

Parity	Nulliparous	3 (8.1)	3 (8.6)	0.77^*∗∗*^
	1–3 children	26 (70.3)	22 (62.9)	
	4–7 children	8 (21.6)	10 (28.6)	

LKR = Sri Lankan rupees (150LKR = 1USD). Living with others includes parents, siblings, friends, or relatives. Primary education = grade 5–10; secondary education = GCE ordinary level. ^*∗*^Groups were compared with the independent sample *t*-test. ^*∗∗*^Groups were compared with chi-square test of independence.

**Table 2:** Comparison of mean scores of health-promoting behaviors and menopausal symptoms scores between experimental and control groups in three stages of evaluation (*n* = 72).

Parameter	Group	Evaluations			Within-group comparison (*p* value)^*∗*^	Between-group comparison (*p* value)^*∗*^	Between-group comparison at the end of 6-month follow-up (*p* value)^*∗∗*^
		Before the intervention, mean (SD)	Immediately after the intervention, mean (SD)	After 6-month follow-up, mean (SD)			
*Health-promoting behaviors*							
Health responsibility	E	18.08 (4.02)	21.70 (1.50)	27.78 (0.67)	<0.001	<0.001	<0.001
	C	17.34 (1.78)	18.05 (1.76)	15.02 (1.80)	<0.001		
Physical activities	E	14.83 (2.12)	20.29 (1.72)	23.62 (1.51)	<0.001	<0.001	<0.001
	C	13.08 (1.31)	12.77 (1.35)	15.82 (1.29)	<0.001		
Nutrition	E	21.56 (2.64)	22.94 (1.79)	28.00 (0.52)	<0.001	<0.001	<0.001
	C	17.91 (1.68)	18.17 (1.44)	18.20 (1.98)	0.36		
Spiritual growth	E	22.78 (3.21)	23.32 (2.18)	27.86 (0.88)	<0.001	<0.001	<0.001
	C	18.45 (1.88)	18.60 (1.80)	17.51 (2.18)	<0.01		
Interpersonal relations	E	21.35 (3.33)	23.18 (1.72)	27.86 (0.88)	<0.001	<0.001	<0.001
	C	17.71 (2.05)	17.20 (2.15)	17.51 (2.18)	0.07		
Stress management	E	19.10 (3.42)	20.59 (1.93)	24.86 (0.78)	<0.001	<0.001	<0.001
	C	15.48 (1.61)	15.62 (1.29)	16.68 (1.54)	<0.01		
Overall health promoting behavior score	E	117.72 (14.60)	132.05 (8.98)	159.83 (3.89)	<0.001	<0.001	<0.001
	C	100.00 (8.81)	100.62 (8.71)	101.42 (8.80)	<0.01		

*Menopausal symptoms scores*							
Psychological symptoms	E	3.13 (3.03)	3.25 (3.01)	2.24 (2.91)	<0.001	<0.001	<0.001
	C	4.42 (3.77)	5.54 (4.61)	8.85 (4.05)	<0.001		
Somato-vegetative symptoms	E	4.81 (3.47)	4.78 (3.37)	3.43 (3.09)	<0.001	<0.001	<0.001
	C	5.52 (3.10)	6.94 (2.98)	9.80 (2.50)	<0.001		
Urogenital symptoms	E	1.48 (1.81)	1.50 (1.80)	1.05 (1.88)	<0.001	<0.001	<0.001
	C	2.14 (2.10)	2.97 (2.45)	5.62 (2.22)	<0.001		
Overall MRS score	E	9.43 (6.97)	9.40 (6.89)	6.72 (6.55)	<0.001	<0.001	<0.001
	C	12.14 (7.24)	15.45 (8.13)	24.28 (7.25)	<0.001		

Groups: E = experimental; C = control; MRS = Menopause Rating Scale. ^*∗*^Means between and within the group were compared with two-way repeated measures ANOVA. ^*∗∗*^Means between the groups at the end of 6 months were compared with one-way ANCOVA while controlling the baseline characteristics.

**Table 3:** Comparison of changes of AAI, CVDRI, muscle strength, and PP between experimental and control groups in two stages of evaluation (*n* = 72).

Measure	Group	Evaluations		Within-group comparison (*p* value)^*∗*^	Between-group comparison at the end of 6-month follow-up (*p* value)^*∗∗*^	Between-group comparison at the end of 6-month follow-up (*p* value)^*∗∗∗*^
		Before the intervention, mean (SD)	After 6-month follow-up, mean (SD)			
Weight (kg)	E	55.38 (8.99)	52.69 (8.30)	<0.001	0.001	<0.001
	C	59.75 (12.47)	61.55 (12.62)	<0.001		

WC (cm)	E	82.75 (8.09)	79.95 (8.27)	<0.001	<0.001	<0.001
	C	86.65 (11.32)	89.27 (11.65)	<0.001		

HC (cm)	E	96.57 (7.20)	95.34 (7.47)	0.004	0.008	<0.001
	C	100.06 (11.96)	101.73 (11.99)	<0.001		

WHR	E	0.85 (0.04)	0.83 (0.05)	<0.001	0.002	<0.001
	C	0.86 (0.04)	0.87 (0.05)	0.003		

BMI (kg/m^2^)	E	24.69 (3.78)	23.50 (3.55)	0.002	0.001	<0.001
	C	26.07 (4.72)	26.87 (4.87)	<0.001		

SBP (mmHg)	E	121.94 (17.29)	118.83 (17.82)	0.002	0.37	0.06
	C	117.25 (13.98)	122.22 (13.97)	<0.001		

DBP (mmHg)	E	78.00 (10.71)	74.72 (9.57)	0.002	0.04	0.001
	C	76.42 (9.19)	79.00 (8.02)	0.03		

FBS (mg/dl)	E	93.73 (26.29)	77.21 (14.33)	<0.001	<0.001	<0.001
	C	100.80 (36.31)	113.31 (37.97)	0.07		

Total cholesterol (mg/dl)	E	187.62 (43.10)	175.81 (43.54)	0.28	0.08	0.25
	C	183.49 (36.83)	194.62 (46.47)	0.27		

Triglycerides (mg/dl)	E	100.30 (60.05)	80.70 (38.93)	0.12	0.65	0.46
	C	116.58 (57.26)	100.41 (47.72)	0.06		

HGS (kg)	E	15.37 (4.50)	20.48 (4.88)	<0.001	0.001	<0.001
	C	16.40 (5.39)	16.22 (5.07)	0.52		

GS (m/s)	E	1.09 (0.14)	1.53 (0.24)	<0.001	<0.001	<0.001
	C	1.22 (0.18)	0.90 (0.09)	<0.001		

Groups: E = experimental; C = control; WC = waist circumference; HC = hip circumference; WHR = waist to hip ratio; BMI = body mass index; SBP = systolic blood pressure; DBP = diastolic blood pressure; FBS = fasting blood sugar; HGS = hand grip strength; GS = gait speed. ^*∗*^Means within the group were compared with the paired sample *t*-test. ^*∗∗*^Means between the groups after 6-month follow-up were compared with the independent sample *t*-test. ^*∗∗∗*^Means between the groups at the end of 6 months were compared with one-way ANCOVA while controlling the baseline characteristics.

## Data Availability

The data used to support the findings of this study are available from the corresponding author upon request.
